This article has been retracted.

# Drop Height Impacts the Lower Limb Elastic Energy's Utilization for Male High Jumpers: A Experimental Research from Biomechanics

**DOI:** 10.1155/2022/8301477

**Published:** 2022-04-11

**Authors:** Zehao Tong, Wenjia Chen, Hang Xu, Feng Zhai

**Affiliations:** ^1^College of Physical Education, China University of Mining and Technology, Xuzhou 221116, China; ^2^Department of Medical Imaging, Xuzhou Medical University, Xuzhou 221004, China

## Abstract

The study's objective is to clarify the influence of drop height on elastic energy's utilization of the lower extremity, to indicate the correlations between elastic energy's utilization and personal best, and to determine the optimal loading height for elastic energy's utilization for male high jumpers. Ten male athletes who belong to high jump events work out the drop jump at different drop heights (0.3 m, 0.45 m, 0.6 m, and 0.75 m). Two AMTI force platforms were used to capture the dynamics data for the lower extremity. Drop height has obvious influence on utilization ratio for elastic energy (*P* < 0.01). The utilization ratio of elastic energy has no note correlation with personal best (*r* = 0.149, *P* > 0.05). In this study, the optimal loading height for utilization ratio of elastic energy was 0.75 m. The optimal loading height can be determined in terms of the elastic energy utilization ratio for each high jumper to enhance their training effects.

## 1. Introduction

During jumps, muscles undergo a cycle of combined motions which included an eccentric stage and a fast concentric stage. The cycle is termed as “stretch-shortening cycle (SSC).” During this period, the elastic energy is accumulated and released by muscle-tendon complex stretching and shortening. The utilization of elastic energy in the concentric shortening phase lays a solid foundation for sports performance during the stretch-shortening cycle. In this period, the muscle-tendon complex plays the vital role in the energy's utilization [1]. Its full stretch could use the elastic energy and reduce the energy waste in the stretch-shortening cycle.

Previous literatures believed that the utilization of elastic energy is a crucial factor in the study of stretch-shortening cycle. Cavagna and Margaria [2] prove the existence of the utilization of elastic energy in the muscle tendon complex by the animal experiments. Wiesinger et al. observed that the Achilles tendon recovery strain in athletes (represented by ski jumpers and distance runners) whose sport required utilization of elastic energy during stretch-shortening cycle was significantly higher than in controls by using motion capture, ultrasonography, and dynamometry [3]. Konow and Roberts believe that the muscle-tendon complex could store the elastic energy and magnify the power during the stretch shorten cycle [4]. Kopper et al. found that in the range of motion of 40° for knee and ankle joints, the acceleration of gastrocnemius and soleus muscles at their maximum lengths was greater than that at the end of joint flexion and also larger than that at the beginning of joint extension [5]. Waugh et al. found that children could not effectively utilize stored elastic energy when performing vertical hopping at a fixed frequency compared to adults, which was considered as one influencing factor that children's muscle efficiency was significantly lower than that of adults during exercise [6].

Drop jump (DJ), as a typical movement in the stretch-shortening cycle, has been treated as the daily routine for high jumpers in the physical fitness training program. Personalized load arrangement and measurement in special physical fitness training of elite athletes were the prerequisite to improve training effect on them. Optimal loading height is a significant symbol for personalized load arrangement and measurement [7]; it means in this height, the certain parameters is maximal. [8] Researchers have determined the maximum reactive strength index and average power output height for drop jump. Kopper et al. found that in the heights 0.35 cm and 0.5 m, average power output is maximal. Byrne et al. [5] revealed that 0.4 m and 0.6 m are an optimal loading height reactive strength index. Zehao et al. [9] found that at a height of 0.45 m, high jumper's reactive strength index and average power output reached the peak [10]. Di Giminiani and Petricola [11] suggest that athletes need to determine their individual optimal loading height for average power output, in order to control their training process.

High jump requests the maximum takeoff height or the shortest ground contact time during the stretch-shortening cycle. Generally, if the coupling from eccentric stretch to concentric shortening for the muscle-tendon complex is less than 170 ms, the cycle is defined as short-term stretch-shortening cycle and long-term stretch-shortening cycle if greater than 170 ms. [12] In terms of the tread-jump phase during a high jump, the coupling from eccentric stretch to concentric shortening for the muscle-tendon complex was a short-term stretch-shortening cycle [13], which was significantly different from long-term stretch-shortening cycle in sprint and other events [14]. The optimal loading height for high jumpers in follow-up studies should be determined, Because of the uniqueness of high jumper's stretch-shortening cycle. It aims at improving the jumper's elastic energy utilization.

To sum up, many studies found that elastic energy utilization influences the efficacy of the stretch-shortening cycle but does not determine the optimal loading height for high jumpers, according to the elastic energy utilization and does not illustrate the correlations between the personal best (PB) and elastic energy utilization in the drop jump. Research's objective contains the following: (1) to clarify the influence of drop height on elastic energy's utilization of lower extremity, (2) to indicate the correlations between elastic energy's utilization and PB, and (3) to determine the optimal loading height of elastic energy's utilization for male high jumpers. This study's hypothesis contain the following: (1) elastic energy utilization was influenced by different drop heights, (2) optimal loading height for high jumpers has existed at four heights, and (3) elastic energy's utilization has correlation with the personal best for high jumpers.

## 2. Methods

Ten male high jumpers were recruited to participate in the test (with an age of 20.7 ± 2.32 years old, a body mass of 72.33 ± 5.36 kg, a height of 189.3 ± 4.12 cm, an age of 20.7 ± 2.32 years, a training experience of 5.1 ± 1.51 years, and a personal best of 2.065 ± 0.04 m). All research subjects had no history of disease or sports injury within one month, had not consumed alcohol within 48 hours before the test, had not taken any drugs within 24 hours before the test, and had not participated in any sports unrelated to the test.

Prior to test, the subjects were informed of the research purpose and test procedures and signed the informed consent with full understanding of the test procedures. The subjects should jog in ten minutes for warm-up and stretch their low extremity in five minutes, in order to the preparation of the test. The subjects performed drop jump at 0.3 m, 0.45 m, 0.6 m, and 0.75 m, respectively, in order to master the standard action for drop jump several times at four heights increased step by step. Two force platforms (AMTI HPS400600, USA) were used to capture dynamics data during drop jump at a frequency of 1000 Hz [15]. The plyometric training box (Escape Fitness, UK) was 0.2 m away from the edge of the force platforms.

The action phases were determined according to changes in vGRF. Initial contact occurred at the moment when the vGRF exceeded 10 N for the first time, takeoff occurred at the moment when the vGRF was lower than 10 N for the first time, and recontact occurred at the moment when the vGRF exceeded 10 N for the second time after flight. [16] The time from the ground-off to recontact indicates the flight phase *T*_f_. The formula is shown below [17].

(1) $$\begin{array}{c} \text{The flight height refers to the vertical displacement of center of gravity},H_{\text{f}}=\frac{1}{2}g{\left(\frac{T_{\text{f}}}{2}\right)}^{2}\left(m\right). \end{array}$$

The work in the eccentric phase Eneg (DJ) = *W* × H1, and the work in the concentric period Epos = *W* × H2, where *W* represents the body mass, H1 represents the drop height, and H2 represents the flight height [13]; the extra work of vertical jump is by using elastic energykgm = Eneg − Epos [18, 19]:

(2) $$\begin{array}{c} \text{The elastic energy utilization ratio}=\frac{\text{kgm}}{\text{Eneg}}\times 100\%. \end{array}$$

By quadratic polynomial regression analysis, the effects of drop height on the utilization rate of elastic energy were obtained (*P* < 0.05). One-way Repeated Measure Analysis of Variance (ANOVA) was selected to find the difference at four heights (*P* < 0.05). The highest mean was the optimal loading height for utilization rate of elastic energy. By Pearson's test, the correlations between the utilization rate of elastic energy and PB were investigated (*P* < 0.05). The data were processed with SPSS (v. 25.0, IBM, USA).

## 3. Results

The drop height has affected the utilization ratio of elastic energy obviously (*F* = 89.143, *P* = 0) (Table 1 and Figure 1). As the height increased, the utilization ratio of elastic energy (*P* = 0) was also improved. Compared to 0.3 m, the utilization ratio of elastic energy increased significantly at 0.45 m, 0.6 m, and 0.75 m, while it increased significantly at 0.6 m and 0.75 m (*P* = 0) relative to the drop height of 0.45 m. The utilization ratio of elastic energy at 0.75 m was significantly higher than that at 0.3 m, 0.45 m, and 0.6 m (95.84 ± 0.91%). As the utilization ratio of elastic energy at 0.75 m had the highest mean in all groups, so the optimal loading height for utilization ratio of elastic energy was 0.75 m. In Table 2, the utilization ratio of elastic energy (*P* = 0.297) had no significant correlations with personal best.

## 4. Discussion

As the loading height of drop jump increased, the utilization ratio of elastic energy increased significantly. A great deal of evidence can clarify the reason. The posture of the low limbs is vital to the elastic energy utilization. Previous studies believed that the utilization ratio of elastic energy was affected by the range of motion of knee and ankle joints and the force in the eccentric phase. Kopper et al. found that in the SRM group (with a range of motion of 40° for knee and ankle joints), the acceleration of gastrocnemius and soleus muscles at their maximum lengths was greater than that at the end of joint flexion and also greater than that at the beginning of joint extension. There was no difference in the LRM group (with a range of motion of 80° for knee and ankle joints). In the SRM group, a large amount of elastic energy was stored at the end of joint flexion and utilized at the beginning of joint extension [5]. Therefore, this SRM technique also could form the BDJ (bounce drop jump) [20], which pursues the shortest ground contact time during drop jump. The short contact time is another condition of elastic energy utilization. It could reduce the loss of energy, when the contact time is short.

However, the short contact time requires that the low extremity need to resist the high loading impact in the higher drop height to keep the fast muscle contraction. It is precisely that high jump training contained numerous fast takeoffs and full flexion and extension with tremendous impact [10]; it makes the muscle tendon complex absorb the elastic energy in the eccentric phase and utilize them well in the concentric phase with the excessive height (0.75 m). McBride and Snyder found that higher bounce heights were produced in the training group of sprinters and jumpers who performed drop jumps at 40 cm, 60 cm, and 80 cm. The authors believed that the force in the eccentric stage increased promoting the utilization of elastic energy [18]. The vGRF in the eccentric phase was mainly controlled by active muscle contraction, and the preactivation and stretch reflex levels were limited at a higher height, so the active contraction of the low limb was affected. As the loading height of drop jump increased, a greater force was generated in the eccentric phase and the soleus short latency reflex was decreased [21]; the range of low limb joint motion was gradually reduced, which was conducive to the storage of elastic energy in the low limb.

The optimal loading height from this study can be used for periodic intervention [22] or postactivation potentiation (PAP) [23] to improve low limb elastic energy utilization of high jumpers during drop jump and to further improve athletic performance by increasing explosive power. In addition, some developed techniques can be used in the sport performance improvement and injury minimum [24–27].

However, the limitation of the research may lie in the difference in sport performance between experimental samples (including professional athletes, college athletes, and young athletes). It should also be emphasized that the AMTI platform can only be used to capture motions of a single experimental sample indicating that other research subjects need to wait for the test, which may reduce the effect of previous concentrated warm-up. In follow-up studies, the profession athlete must be the subjects. What is more, subjects should be required to warm up successively and get ready when their turn comes. According to experiment order, testers should control the warm-up time for each subjects.

## 5. Conclusions

The result shows that drop height has obvious influence on utilization ratio for elastic energy. The utilization ratio of elastic energy has no correlation with personal best. The optimal loading height can be determined in terms of the elastic energy utilization ratio for each jumper to enhance their training. Two hypotheses that elastic energy utilization was influenced by different drop heights and optimal loading height for high jumpers has existed at four heights were supported. Coaches could find the individual optimal loading height for elastic energy utilization, in order to improve the high jumper's low limb explosive power.

## Figures and Tables

**Figure 1:** Utilization ratio of low limb elastic energy during drop jump with different heights.

**Table 1:** The lower limb biomechanical and reactive strength variables during drop jump with different heights.

	0.3 m	0.45 m	0.6 m	0.75 m
Utilization ratio of elastic energy (%)	90.62 ± 1.66^+#^	93.15 ± 1.34^∗^^#^	94.89 ± 1.05^∗^^+^	95.84 ± 0.91^∗^^+^

Note: ∗ indicates an obvious discrepancy to 0.3 m; + indicates an obvious discrepancy to 0.45 m; # indicates an obvious discrepancy to 0.75 m (*P* < 0.05).

**Table 2:** The result of Pearson's test.

		*r*	*P*
Utilization ratio of elastic energy	PB	-0.169	0.297

## Data Availability

The datasets used and/or analyzed during the current study are available from the corresponding author on reasonable request.
